The article "Long non-coding RNA TUG1 promotes cervical cancer progression by regulating the miR-138-5p-SIRT1 axis" was retracted in 2025. Reasons: plagiarized images; overlap with other authors' work.

# Long non-coding RNA TUG1 promotes cervical cancer progression by regulating the miR-138-5p-SIRT1 axis

**DOI:** 10.18632/oncotarget.18224

**Published:** 2017-05-26

**Authors:** Jie Zhu, Huirong Shi, Huina Liu, Xiaojuan Wang, Fengmei Li

**Affiliations:** ^1^ Department of Gynecology and Obstetrics, The First Affiliated Hospital of Zhengzhou University, Zhengzhou 450052, Henan, China; ^2^ Department of Obstetrics and Gynecology, Zhengzhou Central Hospital, Zhengzhou 450000, Henan, China

**Keywords:** cervical cancer, TUG1, SIRT1, miR-138-5p, Wnt/β-catenin

## Abstract

Increasing evidences showed that long non-coding RNAs (lncRNAs) play vital roles in tumor progression. Recent studies indicated that lncRNA TUG1 was upregulated and promoted tumor processes in several cancers. However, the expression and underlying mechanism of TUG1 in cervical cancer remain unclear. In the present study, we found that TUG1 expression was upregulated in cervical cancer tissues and correlated with advanced clinical features and poor overall survival. TUG1 knockdown suppressed cervical cancer cell growth and metastasis *in vitro* and tumor growth *in vivo*. In addition, our results indicated that TUG1 could act as an endogenous sponge by directly binding to miR-138-5p and suppressed miR-138-5p expression. Furthermore, we found that TUG1 could reverse the inhibitory effect of miR-138-5p on cervical cancer cells processes, which might be involved in the activation of SIRT1, a target gene of miR-138-5p, and activation of Wnt/β-catenin signaling pathway. Taken together, we elucidated that TUG1 might promote cervical cancer malignant progression via miR-138-5p-SIRT1-Wnt/β-catenin signaling pathway axis.

## INTRODUCTION

Cervical cancer (CC) is the third most common cancer in women globally [1]. Although various treatments such as surgery, chemotherapy and radiotherapy have been used for the treatment of CC, the prognosis is still poor with a 5-year survival rate of approximately 40% [2, 3]. Lymph node metastasis and distant metastasis are the main reasons for the unsatisfactory prognosis of CC patients [4]. Therefore, uncovering the underlying mechanism of CC would help us to improve therapeutic strategies for the treatment of CC patients.

Long non-coding RNAs (lncRNAs) are defined as ncRNAs >200 nt in length without protein-coding ability [5]. Increasing evidence reported that lncRNAs exert important functions in differentiation, development, and tumorigenesis [6]. For example, Zhang et al. found that MALAT1 overexpression was associated with clear cell renal cell carcinoma progression and prognosis [7]. Gao et al. showed that lncRNA ZFAS1 was an unfavourable prognostic factor and could promote cell progression by activation of the Notch signaling pathway in glioma [8]. Li et al. found that lncRNA HOTTIP overexpression could increase chemoresistance of osteosarcoma cell via activation of the Wnt/β-catenin signaling [9]. Those studies suggested that lncRNAs could exert critical functions in tumor development and progression. However, the functions and underlying molecular mechanisms of lncRNAs in tumor progression remain largely unknown.

The article "Long non-coding RNA TUG1 promotes cervical cancer progression by regulating the miR-138-5p-SIRT1 axis" was retracted in 2025. Reasons: plagiarized images; overlap with other authors' work.

In the current study, our data showed that lncRNA TUG1 overexpression is a characteristic molecular change in CC and explored the roles of TUG1 on the phenotypes of CC cells both *in vitro* and *in vivo*. Moreover, underlying mechanism revealed that TUG1 could act as ceRNAs to regulate SIRT1 expression by sponging miR-138-5p in CC. Together, our study elucidated the first evidence for the TUG1-miR-138-5p-SIRT1-Wnt/β-catenin signaling pathway axis, shedding new light on the diagnosis and treatment for CC patients.

## RESULTS

### LncRNA TUG1 expression levels are elevated in CC

In this study, we used qRT-PCR to explore the expression of TUG1 in 59 pairs of CC tissues. Our data showed that TUG1 expression in CC tissues was upregulated compared to paired non-tumor tissues (Figure 1A; P<0.05). Furthermore, we explored the relationships between clinicopathologic factors and TUG1 expression. Our data showed that TUG1 overexpression was positively correlated with FIGO stage, depth of cervical invasion and lymphnode metastasis (Figure 1B-1D; P<0.05), but not with other clinicopathologic features (Table 1; P>0.05). In addition, Kaplan-Meier analysis revealed that CC patients with high expression of TUG1 had a poor OS (overall survival) (Figure 1E; P<0.05). These findings suggested that TUG1 was involved in CC carcinogenesis.

**Figure 1:** Relative expression levels of lncRNA TUG1 in cervical cancer **(A)** TUG1 expression was upregulated in cervical cancer tissues. TUG1 expression was measured by qRT-PCR and normalized to GAPDH. **(B-D)** TUG1 expression was significantly higher in patients with advanced FIGO stage, lymph node metastasis and depth of cervical invasion. **(E)** Kaplan-Meier analysis showed that patients with high TUG1 expression had a poor overall survival compared to the low TUG1 expression group. * P<0.05.

**Table 1:** Clinicopathological features and lncRNA TUG1 expression in cervical cancer patients

Clinicopathological features	Total	lncRNA TUG1 expression		*P* *value*
		Low	High	
Age				
<45	24	11	13	0.673
≥45	35	18	17	
Tumor size (cm)				
<4.0	26	14	12	0.522
≥4.0	33	15	18	
Histology				
Squamous	41	19	22	0.514
Adenocarcinoma	18	10	8	
FIGO stage				
Ib∼IIa	21	15	6	0.011
IIb∼IIIa	38	14	24	
Lymph node metastasis				
No	29	21	8	0.000
Yes	30	8	22	
Depth of cervical invasion				
<2/3	25	18	7	0.003
≥2/3	34	11	23	

The article "Long non-coding RNA TUG1 promotes cervical cancer progression by regulating the miR-138-5p-SIRT1 axis" was retracted in 2025. Reasons: plagiarized images; overlap with other authors' work.

### LncRNA TUG1 inhibition suppresses CC cells proliferation and invasion

To investigated the role of TUG1 in CC progression, sh-TUG1 were transfected into HeLa and CaSki cells, and qRT-PCR was used to detect the knockdown efficiency (Figure 2A; P<0.05). We performed CCK-8 assay to determine TUG1 effect on CC cells proliferation ability. We found that TUG1 suppression significantly reduced cell proliferation of HeLa and CaSki cells compared to sh-NC group (Figure 2B; P<0.05). Then, we explored the functions of TUG1 on CC cell cycle and cell apoptosis. Flow cytometric analysis showed that TUG1 knockdown could arrest HeLa and CaSki cells at G0/G1 phase (Figure 2C; P<0.05). Meanwhile, TUG1 knockdown increased cell apoptotic events in HeLa and CaSki cells compared to sh-NC group (Figure 2D; P<0.05). Furthermore, we showed that TUG1 inhibition obviously reduced HeLa and CaSki cells invasion ability compared to sh-NC group (Figure 2E; P<0.05). These data suggested that TUG1 might serve as a tumor oncogene in the development of CC.

**Figure 2:** Effect of lncRNA TUG1 on cervical cancer cell growth and metastasis *in vitro* **(A)** The relative expression levels of TUG1 in HeLa and CaSki cells, transfected with sh-TUG1 or sh-NC, were measured by qRT-PCR and normalized to GAPDH. **(B)** CCK-8 assay was used to explore the cell viability of HeLa and CaSki cells transfected with sh-TUG1 or sh-NC. **(C, D)** Flow cytometry was performed to determine the cell cycle and apoptosis of HeLa and CaSki cells transfected with sh-TUG1 or sh-NC. **(E)** Transwell invasion assay was used to explore the invasion ability HeLa and CaSki cells transfected with sh-TUG1 or sh-NC. * P<0.05.

### LncRNA TUG1 inhibition suppresses CC cell growth *in vivo*

To determine the effect of TUG1 on CC tumorigenesis *in vivo*, we injected HeLa cells transfected with sh-TUG1 into nude mice. Our data revealed that sh-TUG1 cell-derived xenograft tumors grew slowly than sh-NC cell-derived xenograft tumors (Figure 3A; P<0.05). The mean weight of sh-TUG1 cell-derived xenograft tumors was also significantly less when compared with sh-NC cell-derived xenograft tumors (Figure 3B; P<0.05). Moreover, we used qRT-PCR to detect TUG1 expression in tumor tissues. Our data showed that TUG1 expression in sh-TUG1 group was obviously downregulated compared with sh-NC group (Figure 3C; P<0.05). Immunohistochemical analysis for Ki67 and PCNA further indicated that sh-TUG1 could reduce cell proliferation in the CC xenograft (Figure 3D and 3E; P<0.05). Therefore, we demonstrated that TUG1 depletion suppressed CC cell growth *in vivo*.

The article "Long non-coding RNA TUG1 promotes cervical cancer progression by regulating the miR-138-5p-SIRT1 axis" was retracted in 2025. Reasons: plagiarized images; overlap with other authors' work.

**Figure 3:** Effect of lncRNA TUG1 on cervical cancer cell growth *in vivo* **(A)** Tumor growth curves determined after injection of HeLa cells stably transfected with sh-TUG1 or sh-NC. The tumor volume was measured every 7 days after 1 week of injection. **(B)** Images of the xenograft tumors from HeLa cells transfected with sh-TUG1 or sh-NC after 6 weeks. **(C)** The relative expression levels of TUG1 in tumor tissues were detected by qRT-PCR. **(D, E)** Reduced cell proliferation in the cervical cancer cell xenograft after sh-TUG1 treatment, as determined by Ki67 **(D)** and PCNA **(E)** immunohistochemistry * P<0.05.

### TUG1 directly interacts with miR-138-5p

Recently, lots of studies indicated that lncRNA might act as a ceRNA or “molecular sponges” to modulate miRNAs [11]. To determine whether TUG1 has a similar mechanism in CC, we used online software starbase 2.0 to predict miRNA target sites. Bioinformatics showed that miR-138-5p had putative binding site with TUG1 (Figure 4A). We used dual-luciferase reporter assay to explore the interaction between miR-138-5p with TUG1. Our data reported that miR-138-5p mimics reduced luciferase activity of pmirGLO-TUG1-Wt, but not of pmirGLO-TUG1-mut (Figure 4B; P<0.05). In addition, we used the biotin–labeled pulldown system to further determine whether TUG1 could pull down miR-138-5p. QRT-PCR revealed that the expression of miR-138-5p was upregulated in TUG1 pulled down pellet (Figure 4C; P<0.05). In addition, we explored miR-138-5p expression in 30 paired of CC tissues. Our data showed that miR-138-5p expression was drastically downregulated in CC tissues and had an inverse correlation with TUG1 expression (r^2^ =0.3325, Figure 4D and 4E; P<0.05). These data revealed that TUG1 might directly bind to miR-138-5p.

**Figure 4:** Validation of TUG1 as a direct target of miR-138-5p **(A)** The sequences of the predicted miR-138-5p binding site and the TUG1 segments containing the wild type binding site are shown. **(B)** Dual-luciferase reporter assay revealed that miR-138-5p mimics decreased luciferase activity of pmirGLO-TUG1-Wt, but not of pmirGLO-TUG1-mut. **(C)** Detection of miR-138-5p using qRT-PCR in the sample pulled down by biotinylated TUG1 probe. **(D)** miR-138-5p expression in 30 paired of cervical cancer tissues was measured by qRT-PCR. **(E)** The correlation analysis was performed between TUG1 expression and miR-138-5p in cervical cancer tissues. *P<0.05.

### MiR-138-5p inhibitors reverse the effect of TUG1 suppression on CC cells

To explore whether the functions of TUG1 were mediated by miR-138-5p, we transfected miR-138-5p inhibitors into sh-TUG1 transfected HeLa and CaSki cells, qRT-PCR showed that the expression levels of miR-138-5p in sh-TUG1 transfected HeLa and CaSki cells were significantly higher than sh-TUG1 + miR-138-5p inhibitors group or sh-NC group (Figure 5A; P<0.05). CCK-8 assay revealed that HeLa and CaSki cells transfected with sh-TUG1 exhibited a significantly lower cell viability compared with sh-TUG1 + miR-138-5p inhibitors group (Figure 5B; P<0.05). In addition, we found that HeLa and CaSki cells transfected with sh-TUG1 exhibited a lower cell invasion ability compared with sh-TUG1 + miR-138-5p inhibitors group (Figure 5C; P<0.05). Those data suggested that miR-138-5p mediated tumor oncogenic effects of TUG1 on CC cells process.

The article "Long non-coding RNA TUG1 promotes cervical cancer progression by regulating the miR-138-5p-SIRT1 axis" was retracted in 2025. Reasons: plagiarized images; overlap with other authors' work.

**Figure 5:** miR-138-5p inhibitor reverses the inhibitory effects of TUG1 suppression on cervical cancer cells **(A)** The relative expression levels of miR-138-5p in HeLa and CaSki cells, transfected with sh-TUG1 or sh-TUG1+ miR-138-5p inhibitors were determined by qRT-PCR. **(B)** CCK-8 assay indicated miR-138-5p inhibitor could reverse the inhibitory effects of TUG1 suppression on cervical cancer cell proliferation. **(C)** Transwell invasion assay showed miR-138-5p inhibitor could reverse the inhibitory effects of TUG1 suppression on cervical cancer cell invasion. *P<0.05.

### SIRT1 is a target of miR-138-5p and regulated by TUG1

MiR-138-5p has been reported as a tumor suppressor gene in pancreatic cancer by targeting SIRT1 [12]. Thus, we suspected that TUG1 might regulate SIRT1 expression through functioning as a ceRNA. To confirm this hypothesis, we detected the expression of SIRT1 in sh-TUG1 transfected HeLa and CaSki cells. Our data showed that TUG1 suppression significantly inhibited SIRT1 expression both in mRNA and protein levels (Figure 6A and 6B; P<0.05). Furthermore, we transfected miR-138-5p mimics into Wt-TUG1 or Mut-TUG1 overexpressed cells. We found that Wt-TUG1 overexpression upregulated SIRT1 expression, and miR-138-5p mimics could abolish the upregulation of SIRT1 induced by TUG1 overexpression (Figure 6C and 6D; P<0.05). All these data suggested that the regulation of SIRT1 by TUG1 required the activity of miR-138-5p.

**Figure 6:** LncRNA TUG1 functions as a ceRNA of SIRT1 **(A, B)** The SIRT1 expression in sh-NC or sh-TUG1 transfected cervical cancer cells was determined by qRT-PCR **(A)** and western blot **(B)**. **(C, D)** The SIRT1 mRNA and protein expression in Wt or Mut TUG1 overexpressed cervical cancer cells transfected with or without miR-138-5p mimics. *P<0.05.

### TUG1 promotes CC malignant progression through Wnt/β-catenin signaling pathway

Lots of studies reported that SIRT1 play crucial roles in cell process by activation of Wnt/β-catenin signaling pathway [13]. Thus, to further explore the potential mechanism that might be involved in the TUG1 associated with malignant progression of CC, we determined related gene expression of Wnt/β-catenin signaling pathway. Western blot revealed that β-catenin expression, c-myc expression and cyclin D1 expression was significantly reduced while E-cadherin expression was obviously augmented when TUG1 was knocked-donwn in HeLa and CaSki cells (Figure 7). Thus, those data suggested that TUG1 might promote cervical cancer cells progresses by miR-138-5p-SIRT1-Wnt/β-catenin signaling pathway axis (Figure 8).

The article "Long non-coding RNA TUG1 promotes cervical cancer progression by regulating the miR-138-5p-SIRT1 axis" was retracted in 2025. Reasons: plagiarized images; overlap with other authors' work.

**Figure 7:** Effect of lncRNA TUG1 on Wnt/β-catenin signaling pathway in cervical cancer cells Western blot showed that TUG1 inhibition suppressed the β-catenin, cyclin D1 and c-myc expression and induced E-cadherin expression in HeLa and CaSki cells.

**Figure 8:** Diagram depicting the regulation mechanism of TUG1 in the tumorigenesis of cervical cancer

## DISCUSSION

Cervical cancer remains the leading gynecologic malignancy worldwide, and it is without doubt that early detection and treatment could significantly increase their chances of survival [1, 2]. Recent studies showed that lncRNAs play great therapeutic potential for human diseases, including CC. For example, Cao et al. showed that GAS5 was downregulated in CC and associated with advanced tumor progression and poor overall survival [14]. Zhang et al. found that lncRNA ANRIL suppressed CC cells proliferation, migration and invasion by inactivation of PI3K/Akt signaling [15]. Zhang et al. showed that the expression of lncRNA MEG3 was decreased in CC and MEG3 could suppress CC cell proliferation and induce cell apoptosis by regulating miR-21 expression [16]. However, the function and underlying mechanism of lncRNAs in CC remain largely unknown.

Taurine up-regulated 1 (TUG1), a 7598-bp lncRNA that maps to chromosome 22q12.2, was initially detected as up-regulation in taurine treated mouse retinal cells, and was essential for normal photoreceptor development [17]. Recent studies reported that TUG1 was dysregulated expression in multiple cancer types. For example, Sun et al. suggested that lncRNA TUG1 was upregulated in colorectal cancer and promoted colorectal cancer metastasis via epithelial-mesenchymal transition pathway [18]. Huang et al. revealed that lncRNA TUG1 expression was upregulated in hepatocellular carcinoma and promoted cell growth and apoptosis by epigenetically silencing of KLF2 [19]. While, Li et al. found that lncRNA TUG1 acted as a tumor suppressor in human glioma by promoting cell apoptosis [20]. Lin et al. revealed that lncRNA TUG1 was downregulated in non-small cell lung cancer and could regulate CELF1 on binding to PRC2 [21]. However, the function and underling mechanism of TUG1 in CC remain largely unclear. In the present study, our data showed that the expression of TUG1 was upregulated in CC tissues and positively corrected with advanced clinical features of CC patients. Overall survival analysis showed that CC patients with high TUG1 expression had a poor prognosis. Moreover, we determined the roles of TUG1 in CC progression. We found that TUG1 inhibition suppressed CC cell proliferation and invasion. In addition, our results showed that TUG1 inhibition suppressed CC cell growth *in vivo*. Thus, our data suggested that TUG1 could act as an oncogene in the progression of CC.

The article "Long non-coding RNA TUG1 promotes cervical cancer progression by regulating the miR-138-5p-SIRT1 axis" was retracted in 2025. Reasons: plagiarized images; overlap with other authors' work.

Although lots of lncRNAs showed to play critical functions in human malignancy, the underlying mechanisms by which lncRNAs modulate tumor growth remains largely unclear [22]. Recent studies showed that lncRNAs may act as competing endogenous RNAs (ceRNAs) which may downregulate miRNAs expression and activities, subsequently modulating the derepression of miRNA targets at the level of post-transcriptional regulation [23]. For example. Huang et al. showed that lncRNA CASC2 could act as a ceRNA by sponging miR-18a in colorectal cancer [24]. Cui et al. reported that overexpression of lncRNA SNHG1 promoted non-small cell lung cancer progression through inhibition of miR-101-3p and activation of Wnt/β-catenin signaling pathway [25]. Therefore, we hypothesized that TUG1 also targeted miRNAs in CC.

In our study, Bioinformatics showed that miR-138-5p had putative binding site with TUG1. Dual-luciferase assay revealed that TUG1 could directly bind miR-138-5p. Pull-down experiment revealed that the expression of miR-138-5p was increased in TUG1 pulled down pellet. Moreover, we found that miR-138-5p expression was downregulated in CC tissues and had an inverse correlation with TUG1 expression. Moreover, our data revealed that miR-138-5p inhibitor could reverse the function of TUG1 inhibition on CC progression. Thus, these results suggested that TUG1 could act as a sponge of miR-138-5p, TUG1 could therefore directly interact with miR-138-5p to restrain its function. Previous study showed that miR-138-5p could suppress pancreatic cancer progression by targeting SIRT1 [12]. Our data revealed that TUG1 inhibition suppressed the mRNA and protein expression of SIRT1. Furthermore, we found that miR-138-5p overexpression abolished the effects of high SIRT1 expression induced by TUG1 overexpression. All these data indicated that the regulation of SIRT1 in CC by TUG1 required the activity of miR-138-5p.

The article "Long non-coding RNA TUG1 promotes cervical cancer progression by regulating the miR-138-5p-SIRT1 axis" was retracted in 2025. Reasons: plagiarized images; overlap with other authors' work.

Wnt/β-catenin signaling pathway regulates a broad range of cell processes, such as cell proliferation, invasion and differentiation [26]. Recent studies showed that lncRNAs could regulate tumor progression via Wnt/β-catenin signaling pathway [27, 28]. Previous studies reported that SIRT1 playing crucial roles in cell process by activation of Wnt/β-catenin pathway [13]. In our study, western blot showed that the expression levels of c-myc, β-catenin and cyclin D1 were decreased while E-cadherin was increased when TUG1 was suppression in CC cells. Thus, we demonstrated that TUG1 might promote CC progression via miR-138-5p-SIRT1-Wnt/β-catenin signaling pathway axis.

In summary, our study indicated that lncRNA TUG1 acted as a tumor oncogene by promoting malignant processes of cervical cancer. Mechanistically, our results suggest that TUG1-miR-138-5p-SIRT1-Wnt/β-catenin axis may be a novel potential therapeutic application for cervical cancer.

## MATERIALS AND METHODS

### Clinical samples

A total of 59 CC tissues and adjacent non-tumor tissues were obtained from patients with CC at the Department of Gynecology and Obstetrics, The First Affiliated Hospital of Zhengzhou University between April 2010 to March 2011. None of the patients had received chemotherapy or radiotherapy prior to surgery. All samples were confirmed by a senior pathologist and were staged according to the Federation International of Gynecology and Obstetrics (FIGO) staging system for CC. This study was approved by the Ethics Committee of Zhengzhou University. Written informed consent was obtained from all patients. The clinicopathological features are shown in Table 1.

### Cell culture and transfection

CC cell lines HeLa and CaSki were purchased from American Type Culture Collection (ATCC). Cells were maintained in DMEM (Gibco) supplemented with 10% fetal bovine serum (FBS, Gibco) at 37 °C in a humidified incubator of 5% CO_2_.

The shRNAs targeting TUG1 (sh-TUG1) and negative control shRNA (sh-NC) were adopted and synthesized by Genechem (Shanghai). The sh-TUG1 sequences are shown as followed: GGTGGTTGAAAGGAATCCT. MiR-138-5p mimics and miR-138-5p inhibitors were purchased from RiboBio (Guangzhou). HeLa and CaSki cells were transfected with shRNAs, miRNA mimics or miRNA inhibitor using Lipofectamine 2000 reagent according to the manufacturer’s instruction (Life Technologies).

### RNA extraction and quantitative real-time PCR

Total RNA was isolated from tumor tissues and cell lines by Trizol reagent (Invitrogen). cDNA synthesis was performed using PrimeScript RT-polymerase (Takara). Quantitative PCR was performed using the SYBR PrimeScript RT-PCR kit (Takara) and GAPDH mRNA was employed as an endogenous control for mRNA. The specific primers for TUG1 and SIRT1 were purchased from Sangon (Shanghai). The expression of miR-138-5p was determined using TaqMan microRNA assays (Ambion) according to the manufacturer’s instructions. The primers for miR-138-5p and U6 snRNA were purchased from Guangzhou RiboBio. Relative expression levels were calculated as ratios normalized against GAPDH or U6 snRNA. The quantification of gene expression was performed by using the 2^−ΔΔCt^ method. The primer sequences were: TUG1, forward, 5'-CTGAAGAAAGGCAACATC-3', and reverse, 5'-GTAGGCTACTACAGGATTTG-3'; miR-138-5p, forward, 5'-GCTTAAGGCACGCGG-3', and reverse, 5'-GTGCAGGGTCCGAGG-3'; SIRT1, forward, 5'-AAAGGAATTGGTTCATTTATCAGAG-3', and reverse, 5'-TTGTGGTTTTTCTTCCACACA-3'.

The article "Long non-coding RNA TUG1 promotes cervical cancer progression by regulating the miR-138-5p-SIRT1 axis" was retracted in 2025. Reasons: plagiarized images; overlap with other authors' work.

### Cell proliferation assay

Cell proliferation was evaluated using Cell Counting Kit-8 (CCK-8, Dojindo) reagent. Briefly, 2x10^3^ cells were plated in each well of 96-well plates. After incubated for 24 h, 48 h, 72 h and 96 h, respectively, 10 ul of CCK-8 solution was added to each well, and cells were incubated at 37°C for 2 h. The absorbance of each well was measured using a microplate reader (BioTek) at a wavelength of 450 nm. Each experiment was performed in triplicate.

### Flow cytometric analysis

After 48 h transfection, cells were collected and washed with PBS. FACS analysis for apoptosis was done using PE Annexin V apoptosis detection kits (BD Biosciences) after 48 h transfection according to the manufacturer's protocol. Cell cycle analysis was performed adopting propidium iodide cell cycle detected kits (BD Biosciences) according to the manufacturer's protocol. Each experiment was performed in triplicate.

### Tanswell invasion assay

The invasive ability of CC cells was evaluated by Transwell chambers (BD Biosciences). Cells (5×10^4^) suspended in 100 μl serum-free medium were seeded into the upper chamber, and the lower chamber was filled with 20% FBS to induce cells invading through the membrane. Matrigel (Sigma) was added on the upper chamber for invasion assay. After 48 h of incubating at 37°C with 5% CO_2_, cells that passed through the pores were fixed in methanol and stained with 0.1% crystal violet and then counted under microscope. Each experiment was performed in triplicate.

### Western blot

Total protein was extracted from cells using RIPA lysis buffer (Beyotime) supplemented with 1% PMSF (KeyGEN). Equal quantity of total protein samples was separated on 10% SDS-PAGE gels and transferred to PVDF membranes. Blots were incubated overnight at 4°C with primary antibody against SIRT1, β-catenin, cyclin D1, c-myc and E-cadherin (Abcam). When secondary antibody incubation finished (Abcam), the electrochemiluminescence (ECL) kit (Tanon) was used to visualize protein signals. GAPDH (Abcam) was used as internal control.

The article "Long non-coding RNA TUG1 promotes cervical cancer progression by regulating the miR-138-5p-SIRT1 axis" was retracted in 2025. Reasons: plagiarized images; overlap with other authors' work.

### Xenograft mouse model

All BALB/c nude mice (4 weeks old, male) were maintained under pathogen-free conditions and all procedures for the mouse experiments were approved by the Animal Care Committee of Zhengzhou University. For the tumor xenografts experiments, stably expressing control shRNA or sh-TUG1 were subcutaneously injected into either side of flank area of 4-week-old male athymic nude mice (n=4, per group). Tumor growth was examined every week, and tumor volumes were calculated using the equation: length×width^2^×0.5. At 6 weeks post injection, mice were euthanized, and the tumors were excised. Animal experiments were performed with the approval of the Institutional Committee for Animal Research and in conformity with national guidelines for the care and use of laboratory animals.

### Dual-luciferase reporter assay

Human HEK293T cells were co-transfected with 150 ng of either empty, pmirGLO-NC, pmirGLO-TUG1-wt or pmirGLO-TUG1-mut (Sangon). 2 ng of pRL-TK (Promega) were also co-transfected with miR-138-5p mimics or miR-NC into HEK293T cells by using Lipofectamie 2000 (Invitrogen). After transfected for 48 h, the luciferase activities were assessed using a dual-luciferase reporter assay kit (Promega), the relative luciferase activity was normalized to Renilla luciferase activity. Each experiment was performed in triplicate.

### Pull down assay with biotinylated miRNA

Cells were transfected with Biotinylated TUG1 or biotinylated NC (RiboBio) using Lipofectamine 2000. The final concentration of each biotinylated miRNA was 20 nM. The cell lysates were collected 48 h after transfection and incubated with M-280 streptaviden magnetic beads (Invitrogen) as described previously [10]. The bound RNAs were purified using TRIzol reagent for further qRT-PCR analysis.

### Immunohistochemical staining

CC xenograft tissues were fixed with 4% PFA and then paraffined. 5 μm thick sections were deparaffinized with xylene and treated with decreasing concentrations of ethanol for hydration. Antigen retrieval was carried out by high pressure boiling of tissue sections in sodium citrate buffer at pH 6.0. Endogenous peroxidase activity was blocked using 0.3% hydrogen peroxide in methanol. After that, tissue sections were blocked with 5% BSA, and incubated with primary antibodies against PCNA and Ki67 (Abcam) overnight at 4°C in a humidified chamber. After incubation with biotinylated secondary antibody, immunohistochemical stainings for PCNA and Ki67 were developed with DAB substrate chromogen system (KeyGEN). Finally, hematoxylin was added as a counterstain and tissue sections were dehydrated in increasing concentrations of ethanol. The PCNA and Ki67 positive cells were photographed with Inverted Research Microscope (Leica).

The article "Long non-coding RNA TUG1 promotes cervical cancer progression by regulating the miR-138-5p-SIRT1 axis" was retracted in 2025. Reasons: plagiarized images; overlap with other authors' work.

### Statistical analysis

Data analysis was performed using SPSS version 18.0 software. Data was shown as mean ± SD from at least three separate experiments. Experimental results were assessed using chi-square test, t test or ANOVA as appropriate. Survival analysis was performed using Kaplan–Meier plots and log-rank tests. P<0.05 was considered as statistically significant.
